# Multimodal Feature Fusion Based Hypergraph Learning Model

**DOI:** 10.1155/2022/9073652

**Published:** 2022-05-16

**Authors:** Zhe Yang, Liangkui Xu, Lei Zhao

**Affiliations:** ^1^School of Computer Science & Technology, Soochow University, Suzhou, China; ^2^Provincial Key Laboratory for Computer Information Processing Technology, Suzhou, China; ^3^Provincial Key Laboratory for Intelligent Engineering in Big Data, Suzhou, China

## Abstract

Hypergraph learning is a new research hotspot in the machine learning field. The performance of the hypergraph learning model depends on the quality of the hypergraph structure built by different feature extraction methods as well as its incidence matrix. However, the existing models are all hypergraph structures built based on one feature extraction method, with limited feature extraction and abstract expression ability. This paper proposed a multimodal feature fusion method, which firstly built a single modal hypergraph structure based on different feature extraction methods, and then extended the hypergraph incidence matrix and weight matrix of different modals. The extended matrices fuse the multimodal abstract feature and an expanded Markov random walk range during model learning, with stronger feature expression ability. However, the extended multimodal incidence matrix has a high scale and high computational cost. Therefore, the Laplacian matrix fusion method was proposed, which performed Laplacian matrix transformation on the incidence matrix and weight matrix of every model, respectively, and then conducted a weighted superposition on these Laplacian matrices for subsequent model training. The tests on four different types of datasets indicate that the hypergraph learning model obtained after multimodal feature fusion has a better classification performance than the single modal model. After Laplace matrix fusion, the average time can be reduced by about 40% compared with the extended incidence matrix, the classification performance can be further improved, and the index F1 can be improved by 8.4%.

## 1. Introduction 

In the machine learning field, the graph is an important data model. If the research objects have a one-to-one relationship between each other, then they can be solved by an ordinary graph such as social networks, gene data, and web page ranking problems [1]. However, in reality, the objects always have a complicated one-to-many or many-to-many relationship between each other [2]. Taking a reference citation, for example, a thesis can cite multiple papers and can be cited by multiple papers. When solving with ordinary graphs, the multivariate relationship will be forcibly shifted into a binary relationship, simply causing information loss. Thus, a hypergraph–a variant of ordinary graph–emerges [3]. Since hypergraphs can better describe the multivariate information between objects, in recent years, hypergraph-based machine learning has become a research hotspot of the machine learning field and has obtained good effect in object segmentation [4], disease diagnosis [5], image classification [6], recommendation system [2, 7], etc.

There are two main methods of using the hypergraph learning model to solve the multivariate relation problem. One method is to extend the hypergraph into an ordinary graph and then use the ordinary graph to solve the hypergraph problems. The representative methods include clique extension, star extension, and line extension [8]. However, in the process of extending a hypergraph to an ordinary graph, the multivariate relation between vertices is changed into a binary relation, which may cause information loss. The other method is to directly aim at the hypergraph structure and its incidence matrix, and solve the optimal hypergraph cut after Laplacian matrix transformation, that is to say, obtain several tangent vectors of the hypergraph Laplacian matrix, and divide the hypergraph into different subsets for classification and clustering. In essence, this is a combinational optimization problem, and the representative methods include the Zhou's normalized Laplacian [3], hypergraph learning regularity optimization [6, 9, 10], hypergraph multimodal structure [11], and hypergraph deep learning [12]. Such methods directly carry out Laplacian transformation and solving on the hypergraph incidence matrix, preventing information loss due to structural transformation. However, all of them are based on one feature extraction method to build a single modal hypergraph structure. If the feature extraction method is not capable enough to fully reflect the relation between objects, it will lead to low-quality hypergraph building and its incidence matrix, finally affecting the performance of the hypergraph learning model.

Therefore, this paper proposed a multimodal feature fusion method, using incidence matrix extension and Laplacian matrix fusion to improve the model performance. The specific work and innovations include the following conditions.

1. When building a hypergraph, first, a single modal hypergraph structure is built based on different feature extraction methods, then different models of hypergraph Laplacian matrices and their weight matrices are extended, and the extended multimodal Laplacian matrices receive model training. The test results show that the extended multimodal incidence matrix could effectively improve the classification performance of the hypergraph learning model.
2. If the dimension of the multimodal incidence matrix obtained by matrix extension is high, it will lead to high computational cost. Therefore, the Laplacian matrix fusion method is put forward, which firstly performs Laplacian matrix transformation on the hypergraph incidence matrix and weight matrix of every model, respectively, and then, these Laplacian matrices are weighted accumulated for further model training. The test results indicate that the Laplacian matrix fusion method can not only reduce the computational cost of the multimodal incidence matrix but also improve the model performance.

## 2. Related Work

Since Zhou et al. firstly proposed the hypergraph learning model [3] and used the “Markov random walk” idea to explain the model, in recent years, there are mainly two approaches to solving multivariate relation problems with the hypergraph learning model: extension method and segmentation method.

The extension method is to expand the hypergraph into an ordinary graph and then use the ordinary graph method to solve the hypergraph problem. Zien firstly raised the star extension approach [13], introducing a new node to every hyperedge of hypergraphs, in which the new node is connected to every vertex of hyperedge by an edge. This approach does not take into account the connection relationship between vertexes within the same hyperedge. Afterwards, Agarwal puts forward a clique extension approach [14], considering every hyperedge as a fully connected subgraph. Although the relationship between vertexes within the same hyperedge is built, it still cannot comprehensively express the connection information of vertexes between hyperedges [12, 15]. To further reduce the information loss during extension, Yang et al. proposed a line extension approach [8] in 2020, considering hyperedges and the nodes within every hyperedge as a new vertex. This approach maximally retains the connection information of vertexes and hyperedges, but it may still bring information loss when dealing with some problems, such as the Fano plane problem [16]. To avoid the information loss problem led by structural transformation, Gao introduced the multimodal concept [11], making different modals correspond to one subhypergraph with weights and training parameters for all subhypergraphs. However, this approach has too many parameters to be optimized, resulting in a high time cost for training. In 2019, Feng proposed the hypergraph Laplacian extension method, which optimized the hypergraph structure while reducing the time cost of machine learning [17]. However, this extension method merely extends the incidence matrix without considering the impact of the weight matrix on the model.

The segmentation method is mainly based on the hypergraph Laplacian matrix to solve the optimal hypergraph cut. Chen et al. applied L2 regularization to optimize the weight parameters of the hypergraph learning model [6, 9]. Chen and Luo used the alternating least square (ALS) method [9] and the coordinate descent method [10] to optimize weight parameters, respectively. Guo utilized the random matrix diffusion idea to optimize the hypergraph Laplacian optimal cut, but this was limited by a single hypergraph structure, needed to optimize the additional target function, and had too high time cost [18]. After that, Zhang et al. raised a hypergraph inductive learning model using the category projection matrix to obtain the category label of the sample [19]. Although the time complexity was brought down to a certain extent, not all dataset information was used in model training, so the classification performance was lowered slightly.

Hence, all existing hypergraph model's solving methods have certain restrictions. The extension approach breaks the multivariate relation between objects. The segmentation approach does not break the limitation of a single hypergraph structure but only optimizes the model solving process, easy to bring high time cost. The multimodal feature fusion method proposed in this paper fuses the abstract features of multiple modals by matrix extension and breaks the limitation of a single hypergraph structure. And in model solving, the Laplacian matrix fusion method helps to reduce the time cost and further enhance the model performance.

## 3. Multimodal Feature Fusion Based Hypergraph Model

### 3.1. General Hypergraph Model

Let *G*=(*V*, *E*, *W*) denote a hypergraph, where *V*={*v*_1_, *v*_2_,…*v*_*n*_, } is the vertex set, and *E*={*e*_1_, *e*_2_,…*e*_*m*_, } is the hyperedge set. The hypergraph's every hyperedge *e*_*j*_(1 ≤ *j* ≤ *m*) contains multiple vertexes *v*_*i*_(1 ≤ *i* ≤ *n*), so the hypergraph *G* can be expressed by incidence matrix *H* ∈ *R*^*n*×*m*^, as shown in Figure 1. In *H*, every element *h*(*v*_*i*_, *e*_*j*_) is defined as

(1) $$\begin{array}{c} h\left(v_{i},e_{j}\right)=\left\{\begin{array}{c} 1,\;\;\text{if }v_{i}\in e_{j},\\ 0,\;\;\text{if }v_{i}\;\notin e_{j}. \end{array}\right. \end{array}$$

Every hyperedge *e*_*j*_ is given a positive weight *w*(*e*_*j*_), and *w*(*e*_*j*_) is calculated by the Gaussian kernel method [20]. Where *di*  *s*(*v*_*i*_, *v*_*k*_)(1 ≤ *i*, *k* ≤ *n*) represents the Euclidean distance between vertex *v*_*i*_ and *v*_*k*_, and *σ* represents the average of the distances between all vertexes.

(2) $$\begin{array}{c} w\left(e_{j}\right)=\sum_{v_{i},v_{k}\in e_{j}}\exp\left(-\frac{\text{dis}{\left(v_{i},v_{k}\right)}^{2}}{\sigma^{2}}\right). \end{array}$$

The diagonal matrix *W* ∈ *R*^*m*×*m*^ is defined, and the elements in diagonal are the weight of every hyperedge *w*(*e*_*j*_)(1 ≤ *j* ≤ *m*), as shown in the following equation:

(3) $$\begin{array}{c} W=\left[\begin{array}{cccc} w\left(e_{1}\right) & 0 & \cdots & 0\\ 0 & w\left(e_{2}\right) & \ldots & 0\\ \vdots & \vdots & \ddots & \vdots \\ 0 & 0 & 0 & w\left(e_{m}\right) \end{array}\right]. \end{array}$$

In the hypergraph, the degree *d*(*v*_*i*_) of every vertex *v*_*i*_ is defined as shown in the following equation:

(4) $$\begin{array}{c} d\left(v_{i}\right)=\sum_{j=1}^{m}w\left(e_{j}\right)h\left(v_{i},e_{j}\right). \end{array}$$

The degree *δ*(*e*_*j*_) of hyperedge *e*_*j*_ is defined as the number of vertexes included in this hyperedge, as shown in the following equation:

(5) $$\begin{array}{c} \delta \left(e_{j}\right)=\sum_{i=1}^{n}h\left(v_{i},e_{j}\right). \end{array}$$

Two diagonal matrix *D*_*v*_ ∈ *R*^*n*×*n*^ and *D*_*e*_ ∈ *R*^*m*×*m*^ is defined. Similar to equation (3), their diagonal elements are the degree of every vertex *d*(*v*_*i*_) and the degree of every hyperedge *δ*(*e*_*j*_) in the hypergraph.

The regularity optimization target function of the hypergraph learning model is shown in the following equation [6, 9]:

(6) $$\begin{array}{c} \arg\;\underset{F}{\min}\;\Phi \left(F\right)≔\Omega \left(F\right)+\lambda \theta \left(F\right)+\mu {\left\|W\right\|}^{2}, \end{array}$$

where *λ* and *μ* are regularization parameters, to balance each item of equation (6). For a *c* classification problem, *F* ∈ *R*^*n*×*c*^ is the eventually solved tangent vector matrix, including the predicted sample category information. *Y* ∈ *R*^*n*×*c*^ is the vector containing real sample labels. In case the vertex *v*_*i*_ falls into the *k*(0 ≤ *k* ≤ *c*) category, then *Y*(*v*_*i*_)[*k*]=1, *Y*(*v*_*i*_)[*p*]=0(0 ≤ *p* ≤ *c* *p* ≠ *k*). *θ*(*F*) is the experience loss function, and Ω(*F*) is the standard loss function, see definitions in the following equations:

(7) $$\begin{array}{c} \theta \left(F\right)={\left\|Y-F\right\|}_{2}^{2}, \end{array}$$

(8) $$\begin{array}{c} \Omega \left(F\right),\\ =\sum_{\begin{array}{c} v_{i},v_{k}\in e_{j} \end{array}}^{m}\frac{w\left(e_{j}\right)h\left(v_{i},e_{j}\right)h\left(v_{k},e_{j}\right)}{\delta \left(e_{j}\right)}\left(\frac{F^{2}\left(v_{i}\right)}{d\left(v_{i}\right)}-\frac{F\left(v_{i}\right)F\left(v_{k}\right)}{\sqrt{d\left(v_{i}\right)d\left(v_{k}\right)}}\right),\\ =\sum_{k=1}^{n}F^{2}\left(v_{k}\right)\sum_{j=1}^{m}\frac{w\left(e_{j}\right)h\left(v_{i},e_{j}\right)}{d\left(v_{i}\right)}\sum_{i=1}^{n}\frac{h\left(v_{k},e_{j}\right)}{\delta \left(e_{j}\right)}-\;\sum_{\begin{array}{c} v_{i},v_{k}\in e_{j} \end{array}}^{m}\sum \frac{F\left(v_{i}\right)h\left(v_{i},e_{j}\right)w\left(e_{j}\right)h\left(v_{k},e_{j}\right)F\left(v_{k}\right)}{\sqrt{d\left(v_{i}\right)d\left(v_{k}\right)}\delta \left(e_{j}\right)},\\ =F^{T}\left(I-D_{v}^{-1/2}{\text{HWD}}_{e}^{-1}H^{T}D_{v}^{-1/2}\right)F,\\ =F^{T}LF. \end{array}$$

In equation (8), *L* is the hypergraph standardization Laplacian matrix.

(9) $$\begin{array}{c} L=I-D_{v}^{-1/2}{\text{HWD}}_{e}^{-1}H^{T}D_{v}^{-1/2}. \end{array}$$

In equation (8), only if two vertexes *v*_*i*_ and *v*_*k*_(*k* ≠ *i*) are at the same hyperedge, it is required to make their standardized labels *F*(*v*_*i*_)/*d*(*v*_*i*_) and *F*(*v*_*k*_)/*d*(*v*_*k*_) to be similar as possible, so that the vertex label can be predicted more accurately. If the hypergraph has degenerated to ordinary graph, then *D*_*e*_ is degenerated to 2*I*, and it is obtained from equation (10) that the relationship between hypergraph's Laplacian matrix *L* and ordinary graph's Laplacian matrix *L*_*A*_ is 1/2 coefficient, in which A represents the adjacent matrix of an ordinary graph.

(10) $$\begin{array}{c} L=I-D_{v}^{-1/2}{\text{HWD}}_{e}^{-1}H^{T}D_{v}^{-1/2},\\ =I-\frac{1}{2}D_{v}^{-1/2}{\text{HWH}}^{T}D_{v}^{-1/2},\\ =I-\frac{1}{2}D_{v}^{-1/2}\left(D_{v}+A\right)D_{v}^{-1/2},\\ =\frac{1}{2}\left(I-D_{v}^{-1/2}AD_{v}^{-1/2}\right),\\ =\frac{1}{2}L_{A}. \end{array}$$

In equation (6), the variables in the optimization target function to be determined are *W* and *F*. Because the target function (6) alone is a convex function relative to *W* and *F*, so it is feasible to use the ALS method [9] and coordinate descend method [10] to optimize *W* and *F*.

In the case of using ALS, it is first to fix *W*, let *δ* Φ(*F*)/*δF*=0, then *F* is optimized.

(11) $$\begin{array}{c} F={\left(I+\frac{1}{\lambda }L\right)}^{-1}Y. \end{array}$$

Second, fix *F* and optimize *W*. By letting *δ* Φ(*W*)/*δW*=0, *W* can be updated as

(12) $$\begin{array}{c} W=\max\left(\frac{F^{T}D_{v}^{-1/2}HI_{\theta }D_{e}^{-1}H^{T}D_{v}^{-1/2}F}{2\mu },0\right). \end{array}$$

Third, repeat the above two steps until *W* and *F* tend to be stable.

In the case of using the coordinate descending method, in each iteration process, two values *W*_*j*_ and *W*_*k*_ should be selected from *W* for updating, and such updating shall be conducted under the constraint conditions of (13), while limiting ∑_*i*=0_^*n*^*W*_*i*_=1. *W*_*j*_^*∗*^ and *W*_*k*_^*∗*^ are the values of updated *W*_*j*_ and *W*_*k*_, see updating process in (14). When *W* becomes stable, we finally obtain an *F*, that is, the ultimate label vector, and the category of a vertex *v*_*i*_ corresponds to index(max(*F*(*v*_*i*_))), that is, the subscript of *F*(*v*_*i*_) maximum.

(13) $$\begin{array}{c} \left\{\begin{array}{c} \left[r_{1},r_{2},\ldots r_{n}\right]=F^{T}D_{v}^{-1/2}H,\\ g_{i}=-r_{i}^{2}D_{e}^{-1}\left(i,i\right), \end{array}\right. \end{array}$$

(14) $$\begin{array}{c} \left\{\begin{array}{c} \begin{array}{cc} \begin{array}{c} W_{j}^{*}=0\\ W_{k}^{*}=W_{j}+W_{k} \end{array} & \text{,if }2\mu \left(W_{j}+W_{k}\right)\;+\left(g_{k}-g_{j}\right)\leq 0, \end{array}\\ \begin{array}{cc} \begin{array}{c} W_{j}^{*}=W_{j}+W_{k}\\ W_{k}^{*}=0 \end{array} & ,\text{if }2\mu \left(W_{j}+W_{k}\right)\;+\left(g_{j}-g_{k}\right)\leq 0, \end{array}\\ \begin{array}{cc} \begin{array}{c} W_{j}^{*}=\frac{2\mu \left(W_{j}+W_{k}\right)+\left(g_{k}-g_{j}\right)}{4\mu }\\ W_{k}^{*}=W_{j}+W_{k}-W_{j}^{*}. \end{array} & ,\text{otherwise}, \end{array} \end{array}\right. \end{array}$$

### 3.2. Hypergraph Laplacian Matrix

The N classification problem solved by the hypergraph model is an *N*-path hypergraph cut problem in essence while the solution to *N*-path hypergraph cut is actually the *N* feature vectors [3] of hypergraph Laplacian matrix. Therefore, if Laplacian matrix can describe more globally and in-depth hypergraph structural information, the accuracy of the hypergraph cut will be increased, and the corresponding classifying performance will also be improved. Zhou et al. firstly proposed the hypergraph learning model [1], adopted Markov random walk idea, and analyzed the hypergraph Laplacian matrix from a probability perspective. The results indicate that the target function (6) of the hypergraph learning model is derived through Markov random walk process. The Markov random walk probability of every vertex in the hypergraph shall follow the following rule: given the current position as *v*_*i*_ ∈ *V*, first, choose a hyperedge *e*_*j*_ from all hyperedges relevant to the vertex *v*_*i*_ at a certain probability and then uniformly randomly choose a vertex *v*_*k*_ ∈ *e*_*j*_(*k* ≠ *i*). Equation (15) provides the probability of a hypergraph vertex's Markov random walk, and equation (16) is a matrix expression of the calculation process of equation (15).

(15) $$\begin{array}{c} p\left(v_{i},v_{k}\right)=\sum_{j=1}^{m}w\left(e_{j}\right)\frac{h\left(v_{i},e_{j}\right)}{\delta \left(e_{j}\right)}\frac{h\left(v_{k},e_{j}\right)}{d\left(v_{i}\right)}, \end{array}$$

(16) $$\begin{array}{c} P=D_{v}^{-1/2}{\text{HWD}}_{e}^{-1}H^{T}D_{v}^{-1/2}. \end{array}$$

Let *S* denotes a subset of hypergraph vertex set *V*, *S*^*c*^ is the complementary set of *S*, and a cut of a hypergraph *G* is dividing a hypergraph into two parts *S* and *S*^*c*^. VolS represents the volume of the set *S*, and *∂S* is the set of cut hyperedge, *∂S*={*e*_*j*_ ∈ *E|e*_*j*_*IS* ≠ *ϕ*, *e*_*j*_∩*S*^*c*^ ≠ *ϕ*}. Equations (17) and (18) define the calculation method of Vol*S* and Vol*∂S*.

(17) $$\begin{array}{c} \text{VolS}=\sum_{v_{k}\in S}d\left(v_{k}\right), \end{array}$$

(18) $$\begin{array}{c} \text{VolS }\partial \text{S}=\sum_{e_{j}\in \partial S}w\left(e\right)\frac{\left|e_{j}\cap S\right|\left|e_{j}\cap \partial S\right|}{\delta \left(e_{j}\right)}. \end{array}$$

Equations (19)–(20) prove the stationary distribution of Markov random walk as *π*(*v*_*k*_) [1].

(19) $$\begin{array}{c} \pi \left(v_{k}\right)=\frac{d\left(v_{k}\right)}{\text{VolV}}, \end{array}$$

(20) $$\begin{array}{c} \sum_{i=1}^{n}\pi \left(v_{i}\right)p\left(v_{i},v_{k}\right),\\ =\frac{1}{\text{VolV}}\sum_{i=1,j=1}^{n,m}\frac{w\left(e_{j}\right)h\left(v_{i},e_{j}\right)h\left(v_{k},e_{j}\right)}{\delta \left(e_{j}\right)},\\ =\frac{1}{\text{VolV}}\sum_{j=1}^{m}w\left(e_{j}\right)\sum_{i=1}^{n}h\left(v_{i},e_{j}\right)\frac{h\left(v_{k},e_{j}\right)}{\delta \left(e_{j}\right)},\\ =\frac{1}{\text{VolV}}\sum_{j=1}^{m}w\left(e_{j}\right)h\left(v_{k},e_{j}\right),\\ =\frac{d\left(v_{k}\right)}{\text{VolV}}. \end{array}$$

It can be seen from equations (15)–(16) that the process of Markov random walk conforms to the hypergraph's standard Laplacian operator *L* in equation (9). If *V* is the feature vector of *P*, then *V* is also the feature vector of *L*. The Laplacian matrix can be deemed as the expression of the hypergraph structure after a random walk. The target function of the hypergraph cut is (21), and equations (19)–(23) prove the minimal cut of Markov random walk, that is to say, making the similarity of the edge connecting different clusters to be minimal (the vertex transition probability is the minimum), while the vertex transition probability within the same cluster is maximal and gradually tends to a stably distributed partition. On account of the difficulty in directly solving (21), it is converted to the basic loss function (8) corresponding to (6), that is, argmin Ω(*F*). The solution to argmin Ω(*F*) is the feature vector corresponding to N minimal nonzero eigenvalues of hypergraph Laplacian matrix. Thus, the Laplacian matrix is very critical to the solving of the hypergraph problem.

(21) $$\begin{array}{c} \min\text{NCut}\left(S,S^{c}\right),\\ =\min\text{Vol}\partial S\left(\frac{1}{\text{VolS}}+\frac{1}{{\text{VolS}}^{c}}\right). \end{array}$$

(22) $$\begin{array}{c} \frac{\text{VolS}}{\text{VolV}}=\sum_{v_{k}\in \partial S}\frac{d\left(v_{k}\right)}{\text{VolV}}=\sum_{v_{k}\in V}\pi \left(v_{k}\right), \end{array}$$

(23) $$\begin{array}{c} \frac{\text{Vol}\partial S}{\text{VolV}},\\ =\sum_{e_{j}\in \partial S}\frac{w\left(e_{j}\right)}{\text{VolV}}\frac{\left|e_{j}\cap S\right|\left|e_{j}\cap S^{c}\right|}{\delta \left(e_{j}\right)},\\ =\sum_{e_{j}\in \partial S}\sum_{v_{i}\in e_{j}\cap S}\sum_{v_{k}\in e_{j}\cap S^{c}}\frac{w\left(e_{j}\right)}{\text{Vol}V}\frac{h\left(v_{i},e_{j}\right)h\left(v_{k},e_{j}\right)}{\delta \left(e_{j}\right)},\\ =\sum_{e_{j}\in \partial S}\sum_{v_{i}\in e_{j}\cap S}\sum_{v_{k}\in e_{j}\cap S^{c}}w\left(e_{j}\right)\frac{d\left(v_{i}\right)}{\text{Vol}V}\frac{h\left(v_{i},e_{j}\right)}{d\left(v_{i}\right)}\frac{h\left(v_{k},e_{j}\right)}{\delta \left(e_{j}\right)},\\ =\sum_{v_{i}\in S}\sum_{v_{i}\in S^{c}}\frac{d\left(v_{i}\right)}{\text{Vol}V}\sum_{e_{j}\in S}w\left(e\right)\frac{h\left(v_{i},e_{j}\right)}{d\left(v_{i}\right)}\frac{h\left(v_{k},e_{j}\right)}{\delta \left(e_{j}\right)},\\ =\sum_{v_{i}\in S}\sum_{v_{i}\in S^{c}}\pi \left(v_{i}\right)P\left(v_{i},v_{k}\right). \end{array}$$

### 3.3. Incidence Matrix Extension

According to equation (9), the hypergraph Laplacian matrix is relevant to the hypergraph incidence matrix *H* and weight matrix *W*. Generally, in the construction of hypergraph structure, it is first to extract the vectorization feature of objects, then similar vertexes are connected in the same one hyperedge based on vertex similarity, and finally, the point-edge incidence matrix *H* and weight matrix *W* are used to represent the basic structure of the hypergraph model. The reason that hypergraphs can depict more information than ordinary graphs is the Laplacian matrices *H* and *I* express more relationships between vertices and vertices and between vertices and hyperedges.

According to equation (15), the probability of every vertex's random walk in the hypergraph is calculated based on the hypergraph incidence matrix. In this process, the hypergraph vertexes can fuse more neighborhood information to improve the vertex classification accuracy. Markov random walk is a conductive, reasonable incidence matrix extension that not only makes Markov random walk to contain vertexes' neighborhood information in the process but also has the opportunity to contact farther vertexes for exploring global information, finally obtain a hypergraph Laplacian matrix fusing more global information. After blending different Laplacian matrices *H* together, the originally nonconnected two vertexes are connected again by different short-path combinations, which can achieve the effect of random matrix *P* “diffusion mapping” [19]. Meanwhile, it is possible to discover the geometry with different scales in heterogeneous hypergraph space, and compared to the original space, it can also keep the globality of hypergraph geometry.

Because different feature extraction methods obtain different feature spaces with different corresponding hypergraph structures, so the incidence matrix extension can be considered as the fusion of multimodal feature space. As shown in Figure 2, a single modal hypergraph incidence matrix *H*_*i*_ ∈ *R*^*n*×m^ is built based on the different feature extraction methods, and then, *H*_*i*_ is further blended to obtain the multimodal incidence matrix *H*′=[*H*_1_‖*H*_2_⋯‖*H*_*n*_] ∈ *R*^*k*×(*n* × *m*)^. Hence, the hypergraph vertex probability transition formula can be rewritten as (24), with its matrix expression means as shown in the following equation:

(24) $$\begin{array}{c} p\left(v_{i},v_{k}\right)=\sum_{t=1}^{n}\sum_{j=1}^{m}w\left(e_{j}\right)\frac{h_{t}\left(v_{i},e_{j}\right)}{\delta \left(e_{j}\right)}\frac{h_{t}\left(v_{k},e_{j}\right)}{d\left(v_{i}\right)},\\ P^{\prime }={D^{\prime }}_{v}^{-1/2}H^{\prime }W^{\prime }{D^{\prime }}_{e}^{-1}{H^{\prime }}^{T}{D^{\prime }}_{v}^{-1/2}. \end{array}$$

It can be seen from equation (2) that the calculation of hypergraph weight is mainly affected by intervertex distance, and the sample feature extraction method or intersample similarity calculation method is different, and then, the intervertex distance obtained will be different, so the weight matrix *W*_*i*_ ∈ *R*^*m*×*m*^ obtained from different modals of incidence matrix *H*_*i*_ will be different. To fuse the hyperedge weight information, the different models of weight matrix *W*_*i*_ are also blended to obtain the multimodal weight matrix *W*′=[*W*_1_‖*W*_2_ ⋯ *|*‖*W*_*n*_] ∈ *R*^*k*×(*m* × *m*)^. As shown in Figure 2, substitute *H*′ and *W*′ into (9) to obtain *L*′=*I* − *D*_*v*_^−1/2^*H*′*W*′*D*_*e*_^−1^*H*′^*T*^*D*_*v*_^−1/2^. *L*′ is substituted into target function (6), and the gradient descend method is used to solve. From the test data in Table 3, the matrix extension method can improve the model classification performance to a certain extent. This indicates that the extended multimodal incidence matrix and weight matrix fuse more abstract features, and the corresponding Laplacian matrix *L*′ contains richer information, so the hypergraph cut obtained is more accurate with a better classification effect. However, as matrix extension results in the rapid growth of matrix dimension, *W*′ and *H*′ are expanded *k* times than original matrices *W* and *H*, bringing greater time cost. In the next section, a Laplacian matrix fusion method will be proposed to solve this problem.

### 3.4. Laplacian Matrix Fusion

Figure 3 describes the main process of Laplacian matrix fusion. Different modals of hypergraph structures correspond to different Laplacian matrices. On the basis of building every modal hypergraph incidence matrix *H*_*i*_ and weight matrix *W*_*i*_, we firstly figure out the corresponding Laplacian matrix *L*_*i*_ under each modal and later perform a weighted sum denoted as *L*^″^; that is,

(25) $$\begin{array}{c} L^{\prime \prime }=\sum_{i=1}^{K}L_{i}\cdot r,s.t.r=\frac{1}{K}, \end{array}$$

*K* represents the number of fusion Laplacian matrices, and then, the standardized loss function Ω(*F*) is rewritten as

(26) ΩF,=r2∑g=1,j=1vi,vu∈ejK,mwgejhgvi,ejhgvu,ejδgejFvidgvi−Fvudgvu2,=r∑g=1,j=1vi,vu∈ejK,mwgejhgvi,ejhgvu,ejδgejF2vidgvi−FviFvudgvidgvu,=r∑g=1K∑u=1nF2vk∑j=1mwgejhgvi,ejdvig∑i=1nhgvu,ejδgej −r∑j=1m∑vi,vu∈ejFvihgvi,ejwgejhgvu,ejFvudgvidgvuδgej,=FT∑g=1KI−Dgv−1/2HgWgDeg−1HgTDgv−1/2·rF,=FTL″F.

In Figure 3, the matrix *L*_*i*_ obtained based on each modal hypergraph contains the information of a single modal incidence matrix *H*_*i*_ and weight matrix *W*_*i*_ while the matrix *L*^″^ fuses the matrix *L*_*i*_ under all modals, containing more comprehensive and higher quality information. Same as Section 3.3, the fused matrix *L*^″^ uses the gradient descent method to solve the target function (6) and trains the ultimate model.

## 4. Experiment and Analysis

### 4.1. Experimental Environment

Aiming at the classification problem, the experiment in this paper compared the hypergraph learning model obtained by training with the proposed method with a typical classification model, ordinary graph, and other hypergraph models. The experimental environment is as follows.

#### 4.1.1. Hardware

The experiment was carried out on GPU colony, available resources as CPU 96 Core, GPU 2 Core GeForce_RTX_2080_Ti/2 Core Tesla_v100_ sxM2_32 GB, memory 512 GB, memory space 500 GB. The programming language is Python 3.7.

#### 4.1.2. Parameters

The KNN method was used to build a hyperedge [21], and that is to say, the vertexes included in the hyperedge are the central vertex and K vertexes nearest to it. To ensure variable consistency, the regularization parameters *λ* and *μ* are set as 2; according to the best result of the experiment, the number of vertices contained in the hyperedge is set to 25.

#### 4.1.3. Datasets

To better verify the performance of the proposed model, four different fields of datasets were selected for the experiment, as shown in Table 1.

*Cat & Dog*. Image datasets, sourced from the official website of Kaggle [22], containing images of cats and dogs, are often used for classification tasks.

*Cifar* 10. Image dataset, a typical computer vision dataset for object identification and classification [23], included a total of 10 categories.

*Ctrip*. Text datasets used the hotel comment data of CTRIP in 2018 [24], in which every comment has been labeled with an emotional direction, such as positive comments or negative comments.

*Spambase*. Numerical value data, the spam datasets provided by the official website of UCI [25], is mainly used to identify and classify spam.

#### 4.1.4. Evaluation Metrics

In this paper, the evaluation indexes used are accuracy, precision, recall, and F1, see the calculation formula in (28)–(30). TP represents the number of samples that are actually positive and predicted as positive, FP represents the number of samples that are actually negative but predicted as positive, FN represents the number of samples that are actually positive but predicted as negative, TN represents the number of samples that are actually negative and predicted as negative.

Accuracy refers to the ratio of the prediction samples correctly classified in total samples.

(27) $$\begin{array}{c} \text{Accuracy}=\frac{\text{TP}+\text{TN}}{\text{TP}+\text{TN}+\text{FP}+\text{FN}}\text{.} \end{array}$$

Precision refers to the ratio of the actually positive samples to the samples predicted as positive.

(28) $$\begin{array}{c} \text{Precision}=\frac{\text{TP}}{\text{TP}+\text{FP}}\text{.} \end{array}$$

Recall refers to the ratio of the samples predicted as positive to actually positive samples.

(29) $$\begin{array}{c} \text{Recall}=\frac{\text{TP}}{\text{TP}+\text{FN}}. \end{array}$$

F1 refers to the harmonic mean of precision and recall, which measures the robustness of the classification model.

(30) $$\begin{array}{c} F1=\frac{2\times \text{Precision}\times \text{Recall}}{\text{Precision}+\text{Recall}}. \end{array}$$

### 4.2. Single Modal Hypergraph Model Performance

This section investigates the performance of a single modal hypergraph models built based on different feature extraction methods and provides references for the experiment in Sections 4.3 and 4.4 about which modals should be selected for feature fusion.  Table 2 compares the classification performance of a single modal hypergraph model built based on different feature extraction methods on image dataset Cat & Dog and text dataset Ctrip.

On Cat & Dog datasets, PHA, VGG, and ResNet represent extracted image features by perceptual harsh [26], VGG [27], and ResNet [28] methods. HSIFT and HVGG represent extracting image features by SIFT [29] and VGG methods after the images are preprocessed with a color difference histogram. RVGG represents extracting image features by the VGG method after the images are Soble sharpened to enhance edge information [30]. After using the above-mentioned methods to extract features, the Euclidean distance is applied to calculate the sample similarity. SIFT represents using the key point matching number to denote the similarity between samples, after extracting the features of images' key points with SIFT.

On Ctrip datasets, TF-IDF, LSI, Word2Vec [31], and Doc2vec [32] represent using these methods to extract data features and using Euclidean distance to calculate sample similarity. Jaccard represents using the Jaccard computing method to measure the similarity between text samples. After obtaining the sample similarity, the hyperedge and hypergraph structures are built according to the KNN method.

It is known from Table 2 that, on Cat & Dog image dataset, the classification performance of the hypergraph model built based on the RVGG method is the best, and the model built based on the PHA method has the poorest quality. On the Ctrip text dataset, the model built based on the Doc2vec method is the best, and the model built based on the Jaccard method has the poorest quality. Thus, the single modal hypergraph models built with different feature extraction methods are different in classification ability. Therefore, it is necessary to find a suitable modal combination to perform incidence matrix extension and Laplacian matrix fusion on multimodal feature fusion hypergraphs.

### 4.3. Model Performance under Modal Combination

This section analyzes the impact of different model combinations, incidence matrix extension, and Laplacian matrix fusion on the hypergraph model's classification performance on text and image datasets, as shown in Table 3. In the table, “Poor + Poor/PHA + SIFT” indicates a new model obtained by combining PHA and SIFT modals. According to the results of the table, the single modal hypergraph model built by PHA and SIFT methods has the poorest quality, belonging to a “poor + poor” combination approach. For each dataset, the second combination approach is a modal combination fusing the best quality and the poorest quality, and the third combination approach is a modal combination fusing the two best qualities.

Comprehensively analyzing Tables 2 and 3, when the hypergraph model quality of two models is equivalent, the incidence matrix extension and Laplacian matrix fusion method are beneficial to improve the classification performance of the new model. On Cat & Dog dataset, Table 2 shows that the quality of the PHA or SIFT-based single modal model is the poorest, and Table 3 shows that the performance of the PHA + SIFT combination is better than PHA and SIFT separately. Likewise, the quality of RVGG and HVGG based single modal models is the best in Table 2, and the performance of the RVGG + HVGG combination in Table 3 is higher than RVGG and HVGG separately. However, when two models' model qualities are varied too much, the incidence matrix extension and Laplacian matrix fusion go on improving model performance. As shown in Table 3, the performance of the RVGG + PHA combination model is lower than RVGG, because the PHA-based single modal model quality is the poorest, which will hinder the performance of the fused new model. On Ctrip datasets, the same conclusion is made as well.

According to the data in Table 3, it is also discovered that after combining different models, the performance of models receiving double fusion of incidence matrix extension and Laplacian matrix is better than that obtained by only incidence matrix extension. Thereby, when choosing modal combinations, it is essential to choose single modal hypergraphs with higher and equivalent quality for the combination and then perform incidence matrix extension and Laplacian matrix fusion, to train and obtain high-quality models.

### 4.4. Influence of Modal Quantity

This section investigates the influence of fused modal quantity on hypergraph model performance, as shown in Figure 4. In the figure, the abscissa axis indicates the fused modal quantity, the data at the bottom of the table reflects the model's classification indexes obtained after fusing multiple modals, and the four curves reflect the tendency that the classification indexes increase with modal quantity. Based on the conclusion of Table 3, the single modal combination with higher and equivalent quality can obtain a higher classification performance, so 1–4 modals are selected for fusion, respectively, following a descending order of quality. Therein, on Cat & Dog datasets, the 1–4 of abscissa axes correspond to such four modal combinations as RVGG, RVGG + HVGG, RVGG + HVGG + VGG, and RVGG + HVGG + VGG + Resnet, respectively. On Ctrip datasets, the 1–4 of abscissa axes correspond to such four modal combinations as Doc2vec, Doc2vec + Word2vec, Doc2vec + Word2vec + LSI, and Doc2vec + Word2vec + LSI + TF-IDF. In Figure 4, the growth trend of the four curves shows that after the fused modal number is larger than 2, the model performance basically tends to be stable. Therefore, in the test of Table 4, all models only fuse two optimal modal combinations.

### 4.5. Time Cost

Table 4 compares the classification performance and time cost of the proposed model with the four single modal models with the best quality on four datasets. Considering Spambase datasets are numeric data and do not involve feature extraction operation, the Euclidean distance and cosine distance are used to figure out the intersample similarity, respectively, and obtain two different single modal hypergraph models, and then, the incidence matrix extension and Laplacian matrix fusion are used, respectively, to compare with the classification performance of single modal models. The experimental results in Table 4 indicate that the proposed multimodal feature fusion method can effectively promote the performance of the hypergraph learning model. Although solely using the incidence matrix extension method may result in larger cost time due to the matrix dimension problem, applying the Laplacian matrix fusion method can effectively reduce the model's time cost only slightly higher than the single modal model with the best quality. On the four datasets, the Laplacian matrix fusion can reduce the time cost by 44.2%, 44.6%, 30.3%, and 40.7% than the incidence matrix extension method, with an average reduction of 40% around.

### 4.6. Comparison with Other Models

This section compares the classification performance of the proposed model with other typical machine learning models, such as KNN, SVM, SVM evolutionary model, ordinary graph model [34], hypergraph model CD, hypergraph model Gd, and hypergraph model Feng. SVM evolutionary model uses the evolutionary algorithm to search the SVM variable value, while the variables of the SVM model are the default initial values of the software package. The hypergraph model CD refers to the hypergraph model obtained by solving the target function with the coordinate descending method, corresponding to equations (13)–(14). The hypergraph model Gd refers to the hypergraph model obtained by solving the target function with the gradient descending method, corresponding to equations (11)–(12). Hypergraph learning Feng refers to the model optimized by the incidence matrix proposed by Feng et al. [16]. For the Ctrip text dataset and Cat & Dog image dataset, it is first to extract features by Word2vec and RVGG approaches and then classify these comparison models compared with the proposed model (refer to Table 1 for the data set division of semisupervised model). 70% of the data set division of the classical classification model is a training set.

It can be seen from Figure 5 that the proposed multimodal fused hypergraph learning model has a better classification performance than typical models such as KNN, SVM, and ordinary graph. Both hypergraph model CD and hypergraph model GD models are single modal models built based on a single feature extraction method, with inferior performance than the proposed model. Although the hypergraph model Feng optimizes the incidence matrix, it ignores the information of hyperedge weight, so its effect is poorer than the proposed model. From the comparison in Figure 5, the proposed multimodal feature fusion method, by virtue of matrix extension and Laplacian matrix fusion, breaks the limits of the single hypergraph structure, fuses multimodal abstract features, and promotes the performance of the hypergraph model.

## 5. Conclusion

Existing hypergraph learning models are all single modal models built based on one feature extraction method, with limited feature extraction and abstract expression ability. This paper proposed a multimodal feature fusion method, making the single modal hypergraph structures built based on different feature extraction methods to fuse multimodal abstract features through extending the incidence matrix and its weight matrix. Then, by using the Laplacian matrix fusion method, every modal's incidence matrix and weight matrix receive Laplacian matrix transformation, respectively, and then undertake weighted accumulation for further model training. In this way, not only the model's time cost is reduced but also the model performance is further improved. As the hypergraph neural model is put forward, hypergraph shows its efficient learning ability in the deep learning field. Therefore, the future study will focus on the hypergraph neural network model and its optimization.

## Figures and Tables

**Figure 1:** Hypergraph and incidence matrix. (a) Hypergraph. (b) Incidence matrix.

**Figure 2:** Hypergraph matrix extension (denotes blend operation).

**Figure 3:** Laplacian matrix fusion.

**Figure 4:** Influence of modal quantity on model performance. (a) Cat & Dog dataset. (b) Ctrip dataset.

**Figure 5:** Comparison of model performance. (a) Cat & Dog dataset. (b) Ctrip dataset.

**Table 1:** Test datasets.

Datasets	Datasets type	Total samples	Numbers of samples in training set	Categories
Cat & Dog	Image	2000	200	2
Cifar 10	Image	40000	6000	10
Ctrip	Text	7766	700	2
Spambase	Numerical value	4601	400	2

**Table 2:** Classification performance of single modal hypergraph model.

Datasets	Feature extraction method	Accuracy	Precision	Recall	F1
Cat & Dog	PHA	0.552	0.554	0.574	0.563
	SIFT	0.658	0.660	0.663	0.661
	HSIFT	0.669	0.674	0.678	0.675
	VGG	0.958	0.960	0.957	0.958
	ResNet	0.960	0.961	0.958	0.959
	HVGG	0.963	0.962	0.963	0.962
	RVGG	0.965	0.965	0.965	0.965

Ctrip	Jaccard	0.508	0.505	0.513	0.508
	TF-IDF	0.603	0.609	0.613	0.610
	LSI	0.608	0.612	0.620	0.615
	Word2vec	0.639	0.748	0.651	0.696
	Doc2vec	0.651	0.870	0.657	0.748

**Table 3:** Classification performance of modal combinations.

Datasets	Modal combinations	Incidence matrix extension				Incidence matrix extension & Laplacian matrix fusion			
		Accuracy	Precision	Recall	F1	Accuracy	Precision	Recall	F1
Cat & Dog	Poor + Poor	0.687	0.662	0.674	0.667	0.722	0.718	0.720	0.718
	PHA + SIFT								
	Poor + Good	0.919	0.920	0.919	0.919	0.928	0.926	0.930	0.928
	PHA + RVGG								
	Good + Good	0.975	0.975	0.977	0.976	0.986	0.986	0.986	0.986
	RVGG + HVGG								

Ctrip	Poor + Poor	0.619	0.620	0.619	0.619	0.623	0.621	0.623	0.621
	Jaccard + TF-IDF								
	Good + Poor	0.646	0.821	0.613	0.701	0.648	0.837	0.624	0.711
	TF-IDF + Doc2vec								
	Good + Good	0.659	0.878	0.709	0.785	0.722	0.718	0.720	0.718
	Doc2vec + word2vec								

**Table 4:** Time cost comparison.

Datasets	Model	Accuracy	Precision	Recall	F1	Time (s)
Cat & Dog	RVGG	0.965	0.965	0.965	0.965	20.26
	RVGG + HVGG	0.975	0.975	0.977	0.976	49.04
	Incidence matrix extension					
	RVGG + HVGG	0.986	0.986	0.986	0.986	27.35
	Incidence matrix extension + Laplacian matrix fusion					

Cifar 10	RVGG	0.561	0.570	0.564	0.567	11236
	RVGG + HVGG	0.564	0.573	0.573	0.573	23793
	Incidence matrix extension					
	RVGG + HVGG	0.594	0.613	0.583	0.598	13158
	Incidence matrix extension + Laplacian matrix fusion					

Ctrip	Doc2vec	0.651	0.870	0.657	0.748	59.7
	Doc2vec + word2vec	0.659	0.878	0.709	0.785	106.86
	Incidence matrix extension					
	Doc2vec + word2vec	0.663	0.884	0.721	0.851	74.2
	Incidence matrix extension + Laplacian matrix fusion					

Spambase	Euclidean	0.646	0.701	0.646	0.672	8.17
	Cosin + Euclidean incidence matrix extension	0.654	0.729	0.654	0.689	17.3
	Cosin + Euclidean incidence matrix extension + Laplacian matrix fusion	0.712	0.734	0.696	0.714	10.25

## Data Availability

The data underlying the results presented in the study are available within the article.
